# Evaluation of Incision Margin and Radiotherapy Adjustment in Breast Cancer-Conserving Surgery Based on VR Pathology 3D Reconstruction

This article has been retracted.

**DOI:** 10.1155/2021/2709461

**Published:** 2021-08-16

**Authors:** Li Zhang

**Affiliations:** Zibo Vocational Institute, Zibo 255300, Shandong, China

## Abstract

At present, the incidence of breast cancer is high worldwide and the most effective way to treat breast cancer is surgery. This study mainly explores the application of pathological three-dimensional reconstruction based on VR technology in the evaluation of the margins of breast-conserving surgery and the adjustment of radiotherapy for breast cancer. In the process of making pathological large slices, the slice markers are counted and the upper and outer cutting edges are located and placed in a large embedding box to prevent tissue deformation. ACDSEE6.0 is used to convert the aligned image BMP format into JPG format, the JPG images of each breast are cropped in batches under the same range and size, and then 3DDOCTOR1.0 is imported to edit the images. The boundary edit tool is activated to segment the target area layer by layer to create a boundary data set of the target structure. The stored file is opened and 3D rendering simple surface and volume rendering on the computer is run to display the surface data 3D display and the volume data 3D display. During VR image processing, the data are imported into the VR image workstation and the Radio Dexter software system is used for image adjustment, trimming, and sequence extraction. Then, the preliminary processed CT and MRI data are displayed in pairs. Through multiplane comparison, manual or automatic fusion tools are used to reduce the gap between image sequences. The surgical process is simulated under VR: by changing the window size and viewing angle; using virtual electric drills, cutting tools, and other virtual instruments; ad selecting the operating microscope perspective; and simulating steps such as breast opening, visual field exposure, and tumor resection. The breast tomographic image was reconstructed in multiple planes, and two-dimensional images of any plane could be observed. 10 cases showed high-density shadows and 5 cases showed isodensity shadows. This research contributes to the precise treatment of breast-conserving surgery.

## 1. Introduction

Complete radical mastectomy is accompanied by a large resection area, pain, and breast loss during the operation. Most importantly, pain causes many side effects. Breast cancer is a malignant tumor with a good prognosis, and the survival rate is relatively high compared with other malignant tumors. Therefore, how to improve the quality of life after breast cancer surgery under the premise of improving the survival rate has become the focus of attention. High-frequency color Doppler ultrasound has been routinely used in the diagnosis and differential diagnosis of breast diseases and has great value in the differential diagnosis of benign and malignant breast masses.

Due to the influence of pain, the quality of life after surgery will be greatly reduced, and the incidence of other complications (immune function decline) will be greatly increased. Therefore, effective local cell biopsy reduces the stress response, and safe and effective postoperative analgesia reduces postoperative pain and related complications. VR technology can not only detect most clinically touched or untouched breast masses, but also observe the position of the puncture needle tip in real time during mass puncture. It has been recognized as a safe and effective method. Double breast ultrasound and molybdenum target X-ray radiography are not only economically acceptable, but also easy to operate. SLNB has high accuracy and few complications. The purpose of this study is to explore the correlation between double breast ultrasound and double breast mammography signs and axillary lymph node metastasis, so as to further predict and guide the selection of breast cancer SLNB.

Recently, the concept of wireless augmented and virtual reality (AR/VR) has swept the entire medical world, causing unprecedented interest in academia, industry, and others. Bastug et al. believe that the success of immersive VR experiences depends on solving numerous challenges across multiple disciplines. They used storage/memory, fog/edge computing, computer vision, artificial intelligence, etc. for research. The main requirements of wireless interconnection VR are described, and then some key elements are introduced. In addition, although they have studied three VR case studies and provided numerical results under various storage, calculation, and network configurations, their research method is not logical [1]. Virtual reality immersion (VRI) is an advanced computer-generated technology that reduces subjective reports of pain in procedural medical treatment. Vera et al. believe that VRI reduces brain activity related to pain as measured by functional magnetic resonance imaging. They randomly assigned 24 patients with chronic pruritus (including 16 patients with psoriasis vulgaris caused by dermatitis and eight patients with chronic pruritus due to psoriasis vulgaris) to one who used special goggles or a computer, the screen of the interactive computer game. Before exposure, during exposure, and 10 minutes after exposure, they self-assessed the intensity of itching using a visual analog scale (ranging from 0 to 10). Their research process only selected 24 patients with chronic pruritus, and the number of samples in the study was too small [2]. Mental health issues are inseparable from the environment. Freeman et al. believe that with virtual reality (VR) and computer-generated interactive environments, individuals can repeatedly experience their problematic situations and learn how to overcome difficulties through evidence-based psychotherapy. They conducted a systematic review of empirical research. 285 studies were identified, 86 of which involved evaluation, 45 theoretical developments, and 154 treatments. The main diseases studied were anxiety (*n* = 192), schizophrenia (*n* = 44), substance-related diseases (*n* = 22), and eating disorders (*n* = 18). Although many treatment methods have been identified in their research, the research methods are unreasonable [3]. Freeman et al. believe that the use of virtual reality can promote new learning. They evaluated the delusions and pain of 30 patients with compulsive delusions. The patients were then randomly assigned to virtual reality cognitive therapy or virtual reality, and both were performed in a hierarchical virtual reality social environment for 30 minutes. Although they reassessed their delusional beliefs and real world troubles, their research experiment data are insufficient [4].

This study mainly explores the application of a medical application system based on augmented reality and virtual-reality-based three-dimensional pathological reconstruction based on VR technology in the evaluation of the margins of breast-conserving surgery and the adjustment of radiotherapy. In the process of making pathological large slices, the slice markers are counted and the upper and outer cutting edges are located and placed in a large embedding box to prevent tissue deformation. Use ACDSEE6.0 to convert the aligned image BMP format into JPG format, crop the JPG images of each breast in batches under the same range and size, and then import 3DDOCTOR1.0 to edit the images. Activate the boundary edit tool to segment the target area layer by layer to create a boundary data set of the target structure. Open the stored file and run 3D rendering simple surface and volume rendering on the computer to display the surface data 3D display and the volume data 3D display. During VR image processing, the data are imported into the VR image workstation, and the Radio Dexter software system is used for image adjustment, trimming, and sequence extraction. Then the preliminary processed CT and MRI data are displayed in pairs. Through multiplane comparison, manual or automatic fusion tools are used to reduce the gap between image sequences. Simulate the surgical process under VR : by changing the window size and viewing angle; using virtual electric drills, cutting tools, and other virtual instruments; and selecting the operating microscope perspective, simulate steps such as breast opening, visual field exposure, and tumor resection.

## 2. VR Technology Pathological Three-Dimensional Reconstruction

### 2.1. VR Technology

Based on computer technology, VR integrates graphic resources, digital resources, and other information resources to form interactive visual 3D dynamic vision and tactile animation. The related terminal equipment is used to identify the VR virtual reality scene and bring the experience of the immersion of the real experience to the experiencer. Nowadays, the application of VR technology has a wide range of fields, and it has the advantage of merging with various technologies. For example, the film and television industry, education industry, marketing industry, entertainment industry, and construction industry have become the new preferences of market consumption, gradually forming a new market form. The creative and experiential technology of VR is considered to play an important role in people's future life, bringing new experiences to people's life, work, and study. First, there needs to be a corresponding reference image, and then feature extraction is performed on the corresponding reference image. At the same time, it is necessary to input the images that need to be paired into the data image to collect relevant data. When the feature extraction data values of the two are sufficient, the matching of related feature data is required. After the feature data values are successfully matched, the analysis stage of the parameter model can be carried out [5]. After that, the related image is transformed. After the image is transformed, the sharpness of the image needs to be adjusted to facilitate the user to identify the information. When the sharpness value of the image is adjusted to the best condition, the relevant image can be presented.

In the virtual reality scene, the detailed functions of the 3D model surface are expanded, and the richer the surface details, the higher the performance. However, the richer the detailed functions of the surface are, the more system resources the model occupies. Therefore, in order to provide theoretical support for model mapping, theoretical research on texture mapping is needed. In the virtual reality scene, in order to make the three-dimensional model of the object more realistic, the detailed functions of the surface of the object model are usually very complicated, the number of model grids is greatly increased, and the system delay of most operating resources and other machines related to the same phenomenon occurs. With texture mapping technology, a detailed image with object characteristics can be mapped to the surface of the object, so the object has the detailed characteristics of the image. In other words, a model with a small number of grids shows the characteristics of the model. The number of grids can be increased to reduce the resource consumption of the system and improve the operating speed of the system. In order to prevent erroneous evaluation results due to data interference, a model for a certain period of time is used as the evaluation criterion [6–8].

(1) $$\begin{array}{c} M_{c}=\frac{1}{L}\sqrt{\sum_{i=0}^{l-1}{\left[y\left(L-i\right)-y_{m}\left(L-i\right)\right]}^{2}+y_{m}\left(L-i\right)}, \end{array}$$

where *L* is the evaluation time zone. *E* is the estimated mean square error of the time domain model [9].

(2) $$\begin{array}{c} \text{Crowd}{\left[J\right]}_{d}=\text{Crowd}\left[J\right]+\frac{\text{Crowd}{\left[J+1\right]}_{m}-\text{Crowd}{\left[J-1\right]}_{m}}{f_{m}^{\max}-f_{m}^{\min}}, \end{array}$$

where Crowd[*J*]_*d*_ represents the maintenance target value of MTH. The average square deviation between model estimates is minimized [10].

(3) $$\begin{array}{c} \min\left(M^{2}\right)=\sum_{L=1}^{N}{\left[y^{\prime }\left(L\right)-y\left(L\right)\right]}^{2}\\ =\sum_{L=1}^{N}{\left[y^{\prime }\left(L\right)-\sum_{i=1}^{m}p_{i}F_{i}\left(L\right)\right]}^{2}. \end{array}$$

Among them, *y*(*L*) is the measured value [11]. Data transmission needs to be carried out at all times during the operation.

(4) $$\begin{array}{c} F\left[C\right]=\left(1-\frac{Q_{ppk}}{Q_{H_{1}}}\right)\left(1-\frac{Q_{att}}{2^{l}}\right)\left(1-\frac{Q_{sc}\left(Q_{H_{2}}+Q_{H_{3}}\right)}{2^{l}}\right)\varepsilon . \end{array}$$

*F*[*C*] is the total amount of data transmission. Data loading and transmission require certain information and data support [12].

(5) $$\begin{array}{c} \mathrm{Pr}\left[C_{1}\right]=1-\frac{Q_{sc}\left(Q_{H_{2}}+Q_{H_{3}}\right)}{2^{l}}. \end{array}$$

Among them, Pr[*C*_1_] represents the intensity of data transmission. Information recognition requires the common realization of the same points of each model [13].

(6) $$\begin{array}{c} F_{v}=\left(1-\frac{Q_{ppk}}{Q_{H_{1}}}\right)\left(1-\frac{Q_{att}}{2^{l}}\right)\left(1-\frac{K_{sc}\left(K_{H_{2}}+K_{H_{3}}\right)}{2^{l}}\right)\varepsilon ,\\ F_{M}=\left(1-\frac{Q_{ppk}}{Q_{H_{1}}}\right)\left(1-\frac{Q_{sc}\left(Q_{H_{2}}+Q_{H_{3}}\right)}{2^{l}}\right)\varepsilon , \end{array}$$

*F*_*M*_ represents the final analysis data. The weight coefficient *h*(*i*, *j*) depends on the domain [14].

(7) $$\begin{array}{c} H\left(i,j\right)=\frac{\sum_{k,i}F\left(k,l\right)\omega \left(i,j,k,l\right)}{\sum_{k,j}W\left(i,j,k,l\right)}+E^{\left({\left(t-k\right)}^{2}+{\left(j-i\right)}^{2}/\sigma \right)}. \end{array}$$

Among them, *i* is the pixel index. It takes time to adapt to VR and reality [15].

(8) $$\begin{array}{c} W\left(I,J,k,l\right)=E^{\left(I{\left(I-k\right)}^{2}+{\left(J-l\right)}^{2}/\sigma \right)\times \left({\left(I-k\right)}^{2}/\sigma_{r}^{2}\right)}+F{\left(k,l\right)}^{2}, \end{array}$$

where *k* is a normalized constant. The distance between two or more points in the image can be expressed by Euclidean formula [16].

(9) $$\begin{array}{c} D\left(x,y\right)=\sqrt{{\left(x_{1}-y_{1}\right)}^{2}+{\left(x_{2}-y_{2}\right)}^{2}+\cdots +{\left(x_{n}-y_{n}\right)}^{2}}, \end{array}$$

where *x*_*n*_ is the gray value of the pixel [17].

(10) $$\begin{array}{c} R_{B}=\sum_{i=k+1}^{L}p_{i}. \end{array}$$

The average gray scale of regions *A* and *B* is

(11) $$\begin{array}{c} \phi_{A}=\frac{1}{\lambda }\sum_{i=1}^{k}i*p_{i}=\frac{\phi \left(k\right)}{\lambda \left(k\right)},\\ \phi_{B}=\frac{1}{W}\sum_{i=k+1}^{L}i*p_{i}=\frac{\phi -\mu \left(k\right)}{1-W\left(k\right)}. \end{array}$$

Among them, *ϕ* is the average gray of the whole image.

(12) $$\begin{array}{c} \chi =\sum_{i=1}^{L}i*p_{i}\\ =\psi_{A}\mu_{A}+\psi_{B}\mu_{B}. \end{array}$$

The variance of the two regions is

(13) $$\begin{array}{c} E^{2}=\rho_{A}{\left(\mu_{A}-\mu \right)}^{2}+\rho_{B}{\left(\mu_{B}-\mu \right)}^{2}. \end{array}$$

The virtual surgery system has the advantages of zero risk, repeatable operation, saving educational resources, etc. Experimenters can use it to complete every step from cutting, hemostasis, separation, lesion treatment to suture and can also timely perform every step of the simulation process. The results are analyzed and evaluated, the errors in the operation are corrected, and the various actual situations that emerge in the clinical operation are experienced, and the clinical skills and practical experience are accumulated. These virtual human bodies, virtual organs and tissues can help complete the operation, preoperative planning and simulation of the surgical process, which have great significance for clinical teaching.

### 2.2. Three-Dimensional Reconstruction

The visual and intuitive display after the three-dimensional reconstruction can help the surgeon make a more accurate, in-depth and detailed diagnosis of the disease. Comprehensive three-dimensional imaging of the tumor area can be used to design the incision and resection range of breast-conserving surgery, which further improves the aesthetics after the operation and at the same time further reduces the degree of trauma. At present, the visualization of medical technology is mainly paid more attention in Europe, America, and other countries. The basic principles of 3D reconstruction mainly include level set algorithm and volume rendering ray projection algorithm. In the 3D reconstruction of the surface rendering algorithm, because the reconstructed 3D surface mesh model is usually called the isosurface, the 3D reconstruction process of the surface rendering algorithm is also called the process of isosurface extraction. The isosurface can be understood as having the same combination of gray value pixels [18–20].

(14) $$\begin{array}{c} \left\{\left(x,y,z\right)|f\left(x,y,z\right)=c\right\}. \end{array}$$

Among them, *x*, *y*, and *z* represent the coordinates corresponding to the sampling data points in the three-dimensional space. For the point whose subscript is, its gray value should be [21]

(15) $$\begin{array}{c} Hu\left(i,j,k\right)=\text{scalars}\left(i,+jX+kXY\right). \end{array}$$

Among them, scalars is the head pointer of the input data stream. For the point whose subscript is (*i*,  *j*, *k*), its gray value should be [22]

(16) $$\begin{array}{c} {\text{position}}_{\left(i,j,k\right)}=\left(ia,jb,kc\right). \end{array}$$

### 2.3. Breast Cancer

The various angiogenesis factors produced by breast cancer cells directly stimulate the growth of tumor angiogenesis, resulting in an ultrasound image showing sufficient blood flow in the tumor cells. In addition, under the action of growth-promoting factors secreted by inflammatory cells in breast malignant tumors and surrounding tumor tissues, tumor cells rapidly proliferate and invade surrounding tissues, showing the irregular shape and disordered edges of the tumor in ultrasound images. Moreover, due to the irregularity of the tumor blood vessels, if the tumor grows rapidly, it is easy to cause normal cell pathology and necrosis and insufficient nutrient supply. If the cells undergo necrotic changes during the pathological process, the precipitation of calcium salts in the tissue fluid and other pathological changes are likely to occur due to a series of physiological and biochemical reactions such as cell phagocytosis and decomposition. Therefore, the ultrasound image will show the characteristic attenuation of tiny calcification or cell count. In some studies, the location of the tumor is also a predictor of benign and malignant breast lesions. Breast tumors show different pathological signs according to the type of tissue, reproduction mode, and the response characteristics of surrounding tissues. High-frequency detection is the basis of ultrasound diagnosis of breast diseases and is widely used to determine the size, boundary, shape, internal echo, calcification, and posterior echo of breast tumors. Because primary breast cancer does not invade the basement membrane and surrounding stroma, it is a noninvasive breast cancer, so it does not penetrate the surrounding tissues and has no specific ultrasound characteristics [23, 24].

The effect of chest anesthesia in the past is obvious, and it can completely suppress the pain of chest surgery. However, the surgical process is more complicated, the failure rate of the operation is also high, and the risk of puncture is very high. Once the sympathetic nerve suppression occurs, it will cause a variety of complications and treatment is very difficult. Moreover, the patient's condition after treatment is also very unsatisfactory. The treatment of vertebral nerve block method is one of the earliest clinical applications of traditional neurological diseases. It can completely block the intercostal neuralgia caused by postoperative chest wall incision. However, the previous chest surgery is ideal. In addition to the complexity of spinal nerve block puncture, the technique is more difficult, it is a strict sterility, and relatively high frequency will cause serious complications [25]. Thoracic surgery will cause surgical wounds and a wide range of rib sections. The use of thoracic nerve block technology for pain relief often requires more partial punctures. Obviously, the complexity of puncture and the risk of complications increase. Therefore, in traditional thoracic breast tumor surgery, the actual clinical application of nerve block technology has not yet been popularized [26, 27]. The breast cancer X-ray examination is shown in Figure 1.

When rendering the triangle mesh model, in order to make the display of the model have a certain sense of reality and gloss, it is necessary to calculate the normal vector of the triangle [28]. Assuming that the gradient value of the point (*i*,  *j*, *k*) is (*G*_*i*_, *G*_*j*_, *G*_*k*_), the central difference method using gray value is

(17) $$\begin{array}{c} G_{i}=\frac{0.5\left(Hu_{\left(i+1,j,k\right)}-Hu_{\left(i-1,j,k\right)}\right)}{m},\\ G_{j}=\frac{0.5\left(Hu_{\left(i,j+1,k\right)}-Hu_{\left(i,j-1,k\right)}\right)}{n}. \end{array}$$

When (*i*, *j*, *k*) is the boundary point, the cube whose subscript value differs by 1 may not exist [29].

## 3. Breast-Conserving Surgery Margin Evaluation Experiment for Breast Cancer

### 3.1. Research Objects and Equipment

We selected 16 patients who underwent breast-conserving postoperative whole breast radiotherapy in our department from June 2019 to February 2020. Age was 31–65 years (median age 46 years). Among them, the primary tumor was located in 7 cases on the left side and 9 cases on the right side. All patients signed the informed consent form.

Image sequence scanning equipment includes a 64-slice spiral CT machine (Discovery Ultra, GE) and a 3.0 T magnetic resonance imaging machine (Trio Tim, SIE). The data bearing medium is an ordinary CD disc and the format is DICOM3 format. The data processing equipment is a VR image workstation (Dextroscope, Volume Interaction), including Radio DexterTM1.0 system control platform, VR interactive operation platform, control handle and tracking system, stereo signal transmitter and wireless LCD stereo glasses and other instruments. The 3.0 T magnetic resonance imaging machine and wireless LCD stereo glasses are shown in Figure 2.

### 3.2. Preparation of Continuous Pathological Slices

The excised tumor tissue is stained and marked, the upper cut edge is stained with black ink, and the positioning point is marked by the parallel needle path two-color smear method. Put the marked tissue excised in a refrigerator at −20°C for 3 hours. The purpose is to make the tissue harden after freezing and make it easier to obtain materials. Place the frozen resected tissue specimens on a self-made large sectioning table, with an interval of 3 mm, parallel to the bottom surface of the same thickness, and cut 5–8 layers. Count the slice markers and locate the upper and outer cutting edges, and put them in a large embedding cassette to prevent tissue deformation. The tissue is fixed, gradient dehydrated, transparent, and waxed. After the tissue block is soaked in wax, select the distal surface of the tissue block as the embedding surface, first place the wax model on the embedding table, and inject a sufficient amount of paraffin melt into the wax model. The wax temperature should be higher than the melting point of paraffin wax 2–3°C; then, use clean tweezers to put the tissue into the wax mold. During this process, prevent air bubbles from forming (if there are air bubbles, use tweezers to drive out the air bubbles to ensure that there are no air bubbles on the embedding surface). After the tissue block is laid flat, press the tissue surface evenly with tweezers (ensure that the tissue embedding surface is closely attached to the embedding table). Then put it in cold water to promote coagulation. After the wax block is completely solidified, it will automatically leave the wax mold and float on the water. Use a blade to trim the wax block properly, and leave a 1–2 mm wax edge around the tissue.

### 3.3. 3D Reconstruction Based on 3DDOCTOR

Under the PC (frequency: 3.0 GHz, memory: 5I2 MB, hard disk: 160 GB, resolution: 1024 × 768 pixels), perform three-dimensional reconstruction of the acquired breast data. Since 3DOCTOR1.0 software only allows up to 450 images, 0.2 mm slices can be used to observe the internal structure of the breast.

First use ACDSEE6.0 to convert the aligned image BMP format into JPG format, and then establish a certain action under PHOTOSHOP7.0, crop each breast JPG image in batches under the same range and size, and then import 3DDOCTOR1. 0. Edit the image to form a continuous picture sequence and save it in the IST file format. Use the EDIT/image calibration parameters command to enter the pixel value and layer thickness of each image to set the tomographic parameters.

Use the LabSQL toolkit developed by a free third party. The toolkit integrates multiple modules, which can realize database access using Microsoft ADO and structured query language SQL. Users do not need to perform underlying development and only need to perform simple SQL operations. Easily access a variety of databases such as Access, Oracle, and SQL Server, which are simple and easy to learn, powerful, fast and highly portable, and suitable for most developers.

Activate the boundary edit tool to segment the target area layer by layer to create a boundary data set of the target structure. Enlarge the image; draw the outline of each structure layer by layer; and outline the interface of each image on the breast edges, skin, fat, glands, tumors, tumors, and blood vessels around the tumors.

Open the stored file and run 3D rendering simple surface and volume rendering on the computer to display the surface data 3D display and the volume data 3D display.

### 3.4. Positioning of the Resection Margin of Cancer

For breast cancer surgery, the positioning of the cancer tissue and the human body is very important, and the tumor may be larger, so the positioning of the tumor margin is also very important. The shape of the resected tissue is generally not fixed, but most of it can be represented by a square. This study also uses the square six-sided positioning method to detect the six sides of the resected tissue. The positioning method also uses the real position corresponding to the human body. The patient is in a supine position, and the doctor and the patient are facing each other. The patient's real position is used to define the incisal surface, the patient's upper, lower, front, back, and inner side of the breast. The outer side surface defines the six sides of the cutting edge, which are represented by letters, S = Superior, I = Inferior, A = Anterior, D = Deep, M = Medial, L = Lateral. For cancer tissues that are too large or too small, the square method is not suitable. Select key points and use digital markers to indicate the margins of giant cancer tissues and micro cancer tissues. In Varian Eclipse TPS, the tumor bed volume is delineated by the radiologist on the 3DCT positioning scan image based on the metal clamp at the boundary of the surgical cavity and defined as GTV. GTV was uniformly expanded by 1.0 cm and 1.5 cm to form CTV1 and CTV2; based on the three-dimensional boundary of the tumor removed, CTV3 and CTV4 were uniformly expanded by 1.0 cm and 1.5 cm respectively.

### 3.5. VR Image Processing

Import data: import the data into the VR image workstation and use the Radio Dexter software system for image adjustment, trimming, and sequence extraction.

Sequence fusion: the preliminary processed CT and MRI data are displayed in pairs. Through multiplane comparison, manual or automatic fusion, contrast adjustment, and image range adjustment are used to reduce the gap between image sequences. By shrinking and expanding the field of view, the macro adjustment tool is used to reduce the fusion error of the two sequences again, in order to achieve a seamless connection of the sequences.

Simulate the surgical process under VR: by changing the window size and viewing angle; using virtual electric drills, cutting tools, and other virtual instruments; and selecting the operating microscope perspective, simulate steps such as breast opening, visual field exposure, and tumor resection. Finally, use the voxel editing tool to perform rotation observation and comprehensively evaluate the tumor resection range. Through repeated simulations, judge the precautions and difficulties during the operation.

### 3.6. Surgical Treatment

Breast-conserving surgery plan for breast cancer is tried out by more than two treatment teams. The team members have more than 10 years of experience in breast surgery by the chief surgeon of general surgery, and then the preoperative examination is completed with the assistance of color Doppler ultrasound and radiologists and cooperates with the clinic. The general surgeon's surgical method is formulated. During breast-conserving surgery, sentinel lymph node biopsy and subsequent radiotherapy were performed. Then, according to the postoperative pathological immunohistochemical results, chemotherapy, endocrine therapy, and molecular targeted drug therapy were combined.

## 4. Results and Discussion

### 4.1. Intraoperative, Postoperative, and Pathological Three-Dimensional Reconstruction Margin Evaluation Analysis

Based on the evaluation results of the resection margin of pathological three-dimensional reconstruction, the false negative rate of intraoperative rapid pathological resection evaluation was 6.7% (2/30), and the false negative rate of postoperative routine pathological resection evaluation was 3.4% (1/29).  Table 1 shows the evaluation of the resection margins of patients during operation, after operation, and pathological three-dimensional reconstruction. The pathological tissue section of breast cancer under the microscope is shown in Figure 3.

There was a statistically significant difference between the tumor long diameter *R*1 measured by conventional pathological materials and the tumor long diameter *R*2 measured by pathological three-dimensional reconstruction (*P* < 0.05), and the tumor long diameter *R*2 measured by pathological three-dimensional reconstruction was greater than *R*1. The type of postoperative routine pathology will affect the decision making of adjuvant treatment of breast cancer. Although the two patients in this study did not change the decision of postoperative adjuvant treatment due to the discovery of the components of ductal carcinoma in situ, this result suggests that conventional pathology is selected. Limitations: large slices of more comprehensive pathological types can be found, which can theoretically affect the decision making of postoperative adjuvant treatment. Comparison of tumor length and diameter is shown in Table 2. The tumor structure and cell morphology under light microscope are shown in Figure 4.

The median volumes of CTV1, CTV2, CTV3, and CTV4 are 70.76 (27.54–158.46), 110.11 (38.13–218.54), 23.85 (9.45–111.33), and 38.74 (15.57–162.67) (units are Cubic centimeters). There were statistically significant differences in the volume of CTV1 and CTV3, and CTV2 and CTV4 (all *P* < 0.05). The statistical results are shown in Table 3. The expansion of the three-dimensional boundary of the tumor is shown in Figure 5.

### 4.2. Image Analysis of Breast Cancer Thin Sections

251, 281, 302, 309, 258, 313, 262, 299, 323, 285, 263, 326, 335, 307, 273, 269, and 311 images were obtained by selecting 17 human breast cancer whole breast tomographic images, and 17 images were obtained. (Set of data sets.) Part of the data is shown in Table 4. The analysis of breast cancer infection rate of different images is shown in Figure 6.

In the three-dimensional image, the edge structure of the 5 cases of tumor was observed in the central area of the breast. The tumor can infiltrate into the large breast duct, and the three-dimensional image showed that the edge of the tumor appeared to be cone-shaped and projected below the nipple.  Figure 7 shows the three-dimensional magnetic resonance imaging of the breast under VR technology. The tomographic CT image of the breast is shown in Figure 8.

### 4.3. Vascular Reconstruction around the Tumor

The status of the resection margin is related to the long-term local control of breast-conserving treatment patients. Therefore, it is reasonable to recommend reoperation for patients with positive resection margins and individualized treatment recommendations for patients adjacent to the resection margin. In addition, tumor-related factors including multicenter tumors, tumor histological types, lymphatic involvement, and staging are related to the local control rate of tumors. Limited data show that multicenter tumors defined as multiple lesions in different quadrants have a detrimental effect on local control. However, considering that the rate of local control has increased since multicenter tumors were regarded as a contraindication to breast-conserving surgery, further analysis of this issue in a prospective study may obtain more comprehensive information. When other factors are the same, the local control rate of most histological patients is similar. The evaluation methods of the resection margin during the operation mainly include the gross specimen examination of the tissue removed during the operation and the mammography examination during the operation. For patients with extensive microcalcifications found in preoperative mammography, the metal guidewire can be positioned under X-ray before operation, and the calcified tissues located by the guidewire can be removed during the operation. The margins are first examined by gross specimens, and then the cut tissue block is taken with a molybdenum target to check the distance between the calcification foci and the edge of the tissue to roughly determine the probability of a positive margin. When there is residual calcification at the margin, the probability of a positive margin for pathological detection under microscope is relatively large. The image of blood flow around breast neuroendocrine is shown in Figure 9.

The breast tomographic image is reconstructed in multiple planes, and two-dimensional images of any plane can be observed. According to the penetration of different tissues to the rays, the characteristics of fat, glands, and tumors can be clearly displayed. The fat shadow appears as a gray low-density shadow. The color is slightly white and dense, and tumors also mainly show high-density shadows. Compared with gland imaging, 10 cases show high-density shadows, and 5 cases show isodensity shadows: tumors can be observed with burr sign, lobular sign, etc. Indirect signs or irregular shapes: after enhanced scanning, the tumor shape and edge display in all cases are clearer and the contrast is strong. The tumor characteristics of MSCT tomography are shown in Table 5. The detection rate of each feature of the breast cross section by ultrasound is shown in Figure 10.

## 5. Conclusion

At present, the incidence of breast cancer is high worldwide, and the most effective way to treat breast cancer is surgery. This study mainly explores the application of a medical application system based on augmented reality and virtual reality-based three-dimensional pathological reconstruction based on VR technology in the evaluation of the margins of breast-conserving surgery and the adjustment of radiotherapy. In the process of making pathological large slices, the slice markers are counted and the upper and outer cutting edges are located and placed in a large embedding box to prevent tissue deformation. Use ACDSEE6.0 to convert the aligned image BMP format into JPG format, crop the JPG images of each breast in batches under the same range and size and then import 3DDOCTOR1.0 to edit the images. Activate the boundary edit tool to segment the target area layer by layer to create a boundary data set of the target structure. Open the stored file and run 3D rendering simple surface and volume rendering on the computer to display the surface data 3D display and the volume data 3D display. During VR image processing, the data are imported into the VR image workstation, and the Radio Dexter software system is used for image adjustment, trimming, and sequence extraction. Then the preliminary processed CT and MRI data are displayed in pairs. Through multiplane comparison, manual or automatic fusion tools are used to reduce the gap between image sequences. Simulate the surgical process under VR : by changing the window size and viewing angle; using virtual electric drills, cutting tools, and other virtual instruments; and selecting the operating microscope perspective, simulate steps such as breast opening, visual field exposure, and tumor resection. This research contributes to the precise treatment of breast-conserving surgery. The three-dimensional negative margin width measured by pathological three-dimensional reconstruction has guiding significance for postoperative breast-conserving radiotherapy. The promotion of this study can provide important reference data for the delineation of the target area of the individualized radiotherapy tumor bed after breast-conserving surgery. In future work, this research method can be combined with adjuvant chemotherapy and adjuvant radiotherapy for in-depth research on breast-conserving surgery.

## Figures and Tables

**Figure 1:** Breast cancer X-ray examination (http://alturl.com/pae3i).

**Figure 2:** 3.0 T MRI machine and wireless LCD stereo glasses (http://alturl.com/e4ndk)(http://alturl.com/n359g).

**Figure 3:** The results of intraoperative, postoperative, and pathological three-dimensional reconstruction of the margins.

**Figure 4:** Tumor structure and cell morphology under light microscope (http://alturl.com/ug3fi).

**Figure 5:** Comparison of CTV1 and CTV3, CTV2, and CTV4.

**Figure 6:** Analysis of breast cancer infection rate of different images.

**Figure 7:** Three-dimensional breast magnetic resonance imaging under VR technology (http://alturl.com/ozbyx).

**Figure 8:** Tomographic CT image of the breast (http://alturl.com/t8rvq).

**Figure 9:** Image of blood flow around the breast neuroendocrine (http://alturl.com/429jm).

**Figure 10:** Ultrasonic detection rate of each feature of breast cross section.

**Table 1:** Intraoperative, postoperative, and pathological three-dimensional reconstruction margin evaluation.

Case	Rapid intraoperative pathology	Routine pathology after surgery	Pathological three-dimensional reconstruction
1	Negative	Positive inferior and outer margins	Positive inferior and outer margins
2	Positive inferior and incisional margins	Positive inferior and incisional margins	Positive inferior and incisional margins
3	Positive external margin	Positive upper margin	Positive upper and outer margins
4	Positive after nipple	Positive after nipple	Positive after nipple
5	Negative	Negative	Positive outer margin

**Table 2:** Comparison of tumor length and diameter.

*R*	Median (mm)	Range (m)	*Z*	*P*
*R*1	19.00	10.00–45.00	−2.438	0.015
*R*2	20.00	7.00–49.00		

**Table 3:** Statistical results.

CTV	Median (cm^3^)	Range (cm^3^)	*Z*	*P*
CTV1	70.76	27.54–158.46	−4.372	0.000
CTV2	23.85	9.45–111.33		
CTV3	110.11	38.13–218.54	−4.372	0.000
CTV4	38.74	15.57–162.67		

**Table 4:** Partial data.

Specimen	Layer thickness (mm)	Number of layers	Size (MB)	Resolution (pixels)	Data volume (GB)
CVB-1	0.2	251	34	4064 × 2704	8.53
CVB-2	0.2	281	34	4064 × 2704	9.54
CVB-3	0.2	302	34	4064 × 2704	10.27
CVB-4	0.2	309	34	4064 × 2704	10.51
CVB-5	0.2	258	34	4064 × 2704	8.77
CVB-6	0.2	313	34	4064 × 2704	10.64
CVB-7	0.2	262	34	4064 × 2704	8.91

**Table 5:** MSCT tomography tumor characteristics.

Scan feature	CT manifestations	Invasive ductal carcinoma (*n* = 13)	Invasive lobular carcinoma (*n* = 2)
Flat sweep density	High density	9	1
	Isodensity	4	1
Lump morphology	Round-like	3	2
	Irregular	10	0
Edge feature	Leaf or burr sign	5	0
	Irregular	8	2
Strengthen	Uniform enhancement in the arterial phase	13	2

## Data Availability

The data that support the findings of this study are available from the corresponding author upon reasonable request.
